RETRACTED

# Zoonotic Paramyxoviruses: Evolution, Ecology, and Public Health Strategies in a Changing World

**DOI:** 10.3390/v16111688

**Published:** 2024-10-29

**Authors:** Francesco Branda, Grazia Pavia, Alessandra Ciccozzi, Angela Quirino, Nadia Marascio, Giovanni Matera, Chiara Romano, Chiara Locci, Ilenia Azzena, Noemi Pascale, Daria Sanna, Marco Casu, Giancarlo Ceccarelli, Massimo Ciccozzi, Fabio Scarpa

**Affiliations:** 1 Unit of Medical Statistics and Molecular Epidemiology, Università Campus Bio-Medico di Roma, 00128 Rome, Italym.ciccozzi@unicampus.it (M.C.); 2 Unit of Clinical Microbiology, Department of Health Sciences, “Magna Græcia” University of Catanzaro—“Renato Dulbecco” Teaching Hospital, 88100 Catanzaro, Italy; graziapavia@unicz.it (G.P.); quirino@unicz.it (A.Q.); nmarascio@unicz.it (N.M.); mmatera@unicz.it (G.M.); 3 Department of Biomedical Sciences, University of Sassari, 07100 Sassari, Italy; aciccozzi@uniss.it (A.C.); c.locci3@phd.uniss.it (C.L.); darsanna@uniss.it (D.S.); 4 Department of Veterinary Medicine, University of Sassari, 07100 Sassari, Italy; iazzena@uniss.it (I.A.); npascale@uniss.it (N.P.); marcasu@uniss.it (M.C.); 5 Department of Chemical Physical Mathematical and Natural Sciences, University of Sassari, 07100 Sassari, Italy; 6 Department of Public Health and Infectious Diseases, University Hospital Policlinico Umberto I, Sapienza University of Rome, 00161 Rome, Italy; giancarlo.ceccarelli@uniroma1.it

**Keywords:** emerging zoonotic paramyxoviruses, wildlife–human interface, epidemic potential

## Abstract

The family *Paramyxoviridae* includes a number of negative RNA viruses known for their wide host range and significant zoonotic potential. In recent years, there has been a surge in the identification of emerging zoonotic paramyxoviruses, particularly those hosted by bat species, which serve as key reservoirs. Among these, the genera Henipavirus and Pararubulavirus are of particular concern. Henipaviruses, including the highly pathogenic Hendra and Nipah viruses, have caused severe outbreaks with high mortality rates in both humans and animals. In contrast, zoonotic pararubulaviruses such as the Menangle virus typically induce mild symptoms or remain asymptomatic in human hosts. This review summarizes current knowledge on the evolution, ecology, and epidemiology of emerging zoonotic paramyxoviruses, focusing on recently discovered viruses and their potential to cause future epidemics. We explore the molecular mechanisms underlying host-switching events, viral replication strategies, and immune evasion tactics that facilitate interspecies transmission. In addition, we discuss ecological factors influencing virus emergence, including changes in bat populations and habitats and the role of wildlife–human interfaces. We also examine the public health impact of these emerging viruses, underlining the importance of enhanced surveillance, developing improved diagnostic tools, and implementing proactive strategies to prevent potential outbreaks. By providing a comprehensive overview of recent advances and gaps in knowledge, this review aims to inform future research directions and public health policies related to zoonotic paramyxoviruses.

RETRACTED

## 1. Introduction

In the last decade, emerging and re-emerging infectious diseases, particularly zoonoses, have posed significant challenges to global public health and socioeconomic stability [1,2]. Effective and timely countermeasures often remain elusive, as demonstrated by the Ebola virus outbreak in West Africa, with over 11,000 deaths [3], and the more recent COVID-19 pandemic, which has claimed 7.1 million lives worldwide [4]. In response to emerging growing threats, such as Marburg virus disease, Lassa fever, Crimean–Congo hemorrhagic fever, and Rift Valley fever, the World Health Organization (WHO) has developed a list of priority pathogens with epidemic potential [5,6]. Among the deadliest viral species currently known, zoonotic paramyxoviruses belonging to the *Henipavirus* genus, such as Nipah (NiV) and Hendra (HeV) viruses, warrant close attention [7]. Their primary reservoir is the *Pteropus* fruit bat and both viruses are responsible for severe respiratory and neurological diseases, often fatal, in humans [7]. As of March 2021, Australia had documented 63 cases of natural HeV spillovers in horses, leading to four deaths among seven confirmed human cases [8]. In South Asia, NiV has been linked to zoonotic outbreaks, with case-fatality rates ranging from 70% to 91% [9]. No therapies or vaccinations are available to protect humans against them. In August 2022, a novel shrew-borne henipavirus strain was detected in febrile patients in eastern China, Langya (LayV) virus [10,11]. Infected individuals exhibited moderate symptoms such as fever, cough, nausea, headaches, and fatigue. While the pathogenicity and epidemiological characteristics of LayV are not yet fully understood, its zoonotic potential has raised concerns [12]. Also, at least two zoonotic paramyxoviruses from the *Pararubulavirus* genus, including Menangle (MenV) and Sosuga (SosV) viruses, have been reported to cause moderate illness in humans [13,14,15]. Given the vast diversity of recently identified *paramyxovirus* species circulating within domestic animals, bats, rats, pangolins, squirrels, and shrews, populations characterized by high evolutionary rates and the capacity to cross species barriers, identifying and monitoring those remains a critical priority for future research [16,17,18,19,20]. The increasing overlap between human, animal, and environmental health necessitates an integrated “One Health” approach. This concept recognizes the interconnectedness of human, animal, and ecosystem health, emphasizing that the control of zoonotic diseases like paramyxoviruses requires coordinated efforts across sectors and disciplines to better predict, prevent, and respond to future outbreaks. Moreover, climate changes and several anthropogenic factors could play a pivotal role in viral sharing among previously geographically isolated species, increasing the risk of spillover events [21,22]. To date, the mechanisms by which zoonotic paramyxoviruses overcome cross-species barriers and establish infections in new hosts are not well defined [20,23].

RETRACTED

This review aims to provide a comprehensive overview of the current knowledge on the evolution, ecology, and epidemiology of zoonotic paramyxoviruses, with a focus on recently identified species for which the pathogenic mechanisms remain yet unknown, and their potential to cause future outbreaks. By highlighting the molecular and environmental factors that could influence virus emergence and transmission, this review could guide future research directions and public health policies related to zoonotic paramyxoviruses.

## 2. Evolution of Paramyxoviruses

### 2.1. Genomic and Virological Characteristics

Paramyxoviruses, belonging to the family *Paramyxoviridae*, are a vast group of enveloped single-stranded (ss), unsegmented negative-sense RNA viruses, characterized by a high ability to infect a wide range of host species, including mammals, birds, fish, and reptiles [24]. Their genomic organization includes six to ten open reading frames (ORFs) that encode essential structural and non-structural proteins [25]. All paramyxoviruses share key membrane glycoprotein complexes: the attachment proteins hemagglutinin (H), hemagglutinin-neuraminidase (HN), or glycoprotein (G), defined as the receptor-binding proteins (RBPs), and the fusion (F) protein. The RBPs enable host–receptor binding, to receptors such as proteins or sialic acids, while the F proteins mediate the fusion of the viral envelope with the host cell membrane, enabling viral entry [25]. The nucleocapsid (N) protein contains the viral RNA genome, forming a helical ribonucleoprotein (RNP) complex. This complex serves as the template for viral replication by the RNA-dependent RNA polymerase, which includes the phosphoprotein (P) and the large (L) protein [26,27]. The P gene encodes a variety of accessory proteins through two mechanisms: (i) RNA editing that generates the V, W, and D proteins; and (ii) overlapping ORFs, which produce small basic proteins, termed C proteins [26,27]. Typically, a single G nucleotide insertion results in the synthesis of the V protein, whereas the W and D proteins are derived from mRNAs with two inserted G residues [26,27]. These accessory proteins interfere with the antiviral host’s cellular immune response [28]. The interaction between matrix (M) proteins with N and the membrane-associated glycoproteins plays a critical role in virion assembly [25]. Additionally, some paramyxoviruses, such as those in the *Rubulavirus* genus, possess a small hydrophobic (SH) transmembrane protein alongside the primary structural proteins. Only a subset of paramyxoviruses encodes a fourth integral membrane protein, the transmembrane (TM) protein, which facilitates cell-to-cell fusion but does not contribute to viral entry [29].

RETRACTED

### 2.2. Phylogenetic Classification and Diversity

Currently, the *Paramyxoviridae* family is divided into four subfamilies—*Orthoparamyxo virinae*, *Metaparamyxovirinae*, *Rubulavirinae*, and *Avulavirinae*—encompassing 20 genera and approximately 78 species, based on phylogenetic analysis of the L gene [24]. This genetic differentiation aligns with observed differences in biological, biochemical, and host range characteristics [24]. Among zoonotic paramyxoviruses, avulaviruses primarily infect birds, except the Newcastle disease virus (NDV), which occasionally causes mild, self-limiting infections in individuals in close contact with infected birds [30]. Metaparamyxoviruses exist only as genetic sequences, with no reported isolates to date [27,31], and therefore, they are not considered potential epidemic pathogens. The *Rubulavirinae* subfamily includes the *Orthorubulavirus* and *Pararubulavirus* genera. While pararubulaviruses, such as the MenV and SosV strains, cause relatively mild diseases in humans, their ability to circulate undetected in animal populations and occasionally spill over into humans poses an ongoing public health concern [13,14,32,33].

The *Orthoparamyxovirinae* subfamily represents the largest grouping in the family, including three highly adaptable viral genera: *Morbillivirus*, *Respirovirus*, and *Henipavirus*. Based on the biological characteristics, rapid genetic evolution, moderate-to-severe human illness, and the ever-expanding range of hosts, they have been prioritized for closer consideration over the other genera [34,35,36,37]. Notably, NiV and HeV henipavirus strains represent significant public health threats due to their high mortality rates—ranging from 40% to 90% for NiV—and their capacity for zoonotic transmission [7,8,9]. Although both viruses have demonstrated human-to-human transmission, their relatively low basic reproduction number (R0) reduces the immediate concern over their potential to evolve into highly transmissible agents [7,8,9]. Currently, only the Equivac HeV vaccine for horses, approved in Australia in 2012, is available for preventing Hendra virus infections, mainly due to the need to handle these select agents in biosafety level 4 (BSL-4) laboratories [38]. The identification of Cedar virus, a non-pathogenic henipavirus, provides a promising alternative for research, as it can be studied in laboratories with lower biosafety requirements (BSL-2+) [39]. A newly discovered shrew-borne henipavirus, named LayV, was identified in a febrile patient in eastern China [10,11]. Phylogenetically, it is most closely aligned with Mojiang henipavirus, which was identified in China in 2012 and has been associated with three fatal cases of pneumonia [10,40]. Most recently, Xu and colleagues characterized new henipaviruses from 969 small mammals in Hubei Province, Central China, which shared 68% nucleotide identity with LayV, indicating a significant public health risk [19].

RETRACTED

It is well known that *Rubulavirus*, *Morbillivirus*, and *Respirovirus* genera also encompass several pathogens that are established in humans, such as measles virus (MV), human parainfluenza viruses (HPIVs), and human respiratory syncytial virus (HRSV) [41,42,43]. HPIV-3 and bovine parainfluenza virus 3 (BPIV-3) likely originated in animal hosts before adapting to humans, facilitated by increased human–animal interactions during the domestication of livestock [44]. Similarly, HRSV and bovine respiratory syncytial virus (BRSV) share antigenic and immunopathologic characteristics [45], suggesting potential cross-species transmission events. Notably, MV, a significant human pathogen, is believed to have diverged from rinderpest virus in cattle, with zoonotic transmission occurring around 1000 years ago, coinciding with the rise of large, dense human populations [46]. These zoonotic transitions were likely driven by ecological changes such as the development of agriculture and urbanization, which created new opportunities for viral adaptation to human hosts. These viruses are among the most highly transmissible known, and the recent discovery of significant genetic diversity in wildlife reservoirs raises the question of whether unidentified zoonotic paramyxoviruses from these genera could pose a substantial risk to human health [41,47,48,49,50,51].

The zoonotic paramyxoviruses, hosts, geographical distribution, evolution rate, and their epidemic potential risk are summarized in Table 1.

RETRACTED

### 2.3. Evolutionary Molecular Mechanisms and Implications

The evolutionary pathways of paramyxoviruses are well understood for some species but remain poorly defined for unclassified strains and among subfamilies and genera [23,54,55]. Studies comparing paramyxoviruses with other RNA viruses suggest that they exhibit relatively high rates of cross-species transmission [18], with mutation rates comparable to other RNA viruses [56,57,58]. This heightened capacity for host-switching, along with characteristics such as a non-segmented RNA genome and non-vector transmission, is associated with an increased likelihood of human-to-human transmission following zoonotic spillover [59,60]. A critical question in the emergence of pathogens capable of sustained human transmission (R0 ≥ 1) is whether this is primarily driven by viral adaptation within human hosts or by repeated spillovers of diverse viruses, some of which may already be pre-adapted for human transmission [56]. Woolhouse and colleagues reported that virological traits, such as tissue tropism and transmission routes, affect human transmission rates, and are often conserved among related viruses [61]. As a result, significant adaptive changes would be required to increase R0 in a new host, making pre-adaptation a more likely mechanism in most cases [61]. Each spillover event from an animal reservoir introduces new viral variants into the human population, increasing the likelihood of a virus emerging that can cause an epidemic. Phylogenetic studies across viral families [18,62], and specifically among paramyxoviruses [63], indicate that host-switching between closely related species is a key driver of viral macroevolution. Differences in the replication fitness landscape between these related hosts are sufficient to drive viral adaptation while still allowing for transmission [18,63,64,65]. Orders such as *Chiroptera* (bats) and Rodentia (rats) are particularly suited to amplifying viral diversity and promoting spillover due to their optimized transmission both within and between species. Bats and rodents are recognized as major wildlife reservoirs for paramyxoviruses with unknown zoonotic potential [19,63,66,67].

Previous studies have reported low recombination rates in paramyxoviruses, suggesting that recombination plays a minimal role in the family’s overall evolutionary history [68,69]. McCarthy and Goodman [55], using a larger dataset that included six viral genes and a concatenated multigene analysis, also concluded that recombination is likely not a major driver of evolutionary changes at the family level. Rare recombination events were detected in the H gene of CDV isolates from wild carnivores [70,71]. These findings suggest that although recombination is uncommon, it may contribute to genetic diversity within genera and species, potentially facilitating the emergence of new *paramyxovirus* species.

RETRACTED

Another potential mechanism is “reverse zoonosis”, or anthroponosis, which occurs when pathogens are transmitted from humans to animals. An example of this could be the evolution of CDV, which is thought to have emerged in dogs following cross-species infection with MV from humans. Genetic and evolutionary analyses suggest that CDV, which causes severe disease in domestic and wild carnivores, may have evolved after MV, a closely related morbillivirus, was transmitted from humans to canids, leading to viral adaptation and the emergence of CDV as a distinct pathogen [72]. This case highlights the dynamic nature of Paramyxovirus evolution across species barriers.

The primary evolutionary mechanisms involved in paramyxoviruses spillover to humans are illustrated in Figure 1.

## 3. Ecology and Environmental Factors

### 3.1. Primary Hosts and Natural Reservoirs

Zoonotic paramyxoviruses are maintained in complex ecological networks, where wildlife species play a central role as primary reservoirs. Bats are known to host over 200 different viruses, with RNA viruses showing a higher frequency of spillover [20,66]. This is likely due to the high mutation rates characteristic of several RNA viruses, such as SARS-CoV-2, which caused the recent pandemic, and viruses capable of generating *quasispecies* [57,73,74,75,76]. Such variability may enable rapid adaptation to new host species and shifting environmental conditions, thereby facilitating cross-species transmission [20,66,77,78]. In particular, frugivorous species from the *Pteropodidae* family, genus *Pteropus*, are recognized as the primary reservoirs for several paramyxoviruses, including the highly pathogenic henipaviruses [79]. Bats possess traits that make them highly effective at harboring and spreading zoonotic viruses: their ability to fly allows for long-distance dispersal of pathogens across regions, while their social behavior—such as roosting in large colonies—facilitates viral circulation within populations [22]. Furthermore, bats exhibit a unique immune system that tolerates high viral loads without developing disease, contributing to their role as asymptomatic carriers of paramyxoviruses [80].

NiV is primarily hosted by *P. vampyrus* and *P. hypomelanus* [81,82], prevalent across South and Southeast Asia, while *P. alecto*, *P. poliocephalus*, *P. scapulatus*, and *P. conspicillatus* were identified as natural hosts of HeV [83]. Similar to bats, shrews—insectivores from the family *Soricidae* (Mammalia: *Eulipotyphla*)—harbor a diverse range of viruses, including the recently identified LayV henipavirus [10,11]. A serological study of domestic and wild animals revealed that LayV RNA was primarily detected in shrews, particularly *Crocidura lasiura* and *C. shantungensis*, species commonly found in northeast Asia. The virus was also identified in 5% of dogs and 2% of domestic goats tested, suggesting the possibility of multiple host species, although shrews are suspected to be the natural reservoir [10,11]. Transmission to humans typically occurs via intermediate hosts—horses for HeV, pigs for NiV, and likely domestic animals for LayV—following exposure to infected biological fluids or contaminated fruit [10,11,79]. The role of these intermediate hosts is critical, as they serve as a bridge between the original wildlife reservoirs and human populations. Intermediate hosts can amplify the viral load, increasing the likelihood of transmission to humans through close contact or the consumption of contaminated products. Furthermore, understanding the dynamics of intermediate hosts is essential for identifying potential spillover events and implementing effective surveillance and control measures. This multi-host dynamic complicates efforts to predict and control outbreaks, as spillover can involve a diverse array of species across different ecosystems.

RETRACTED

Avulaviruses are primarily associated with avian species, especially poultry, where they cause significant economic losses due to their highly contagious nature. NDV, part of this group, can infect humans, typically those in close contact with infected birds, such as poultry farmers or workers in live bird markets [30].

Among the pararubulavirus strains, MenV and SosV are notable for their broader host range, including bats, humans, and pigs. MenV was first identified in Australia, where it caused reproductive disorders in pigs and mild flu-like symptoms in humans [13,32]. Unlike other pararubulaviruses, SosV was initially isolated from a wildlife biologist who developed a febrile systemic illness after handling various wildlife species [84]. Phylogenetic analysis and the patient’s history suggested bat origin, which was later confirmed by molecular detection of the virus in *Rousettus aegyptiacus* bats [33].

Respiroviruses, particularly HPIV, are primarily human pathogens; however, zoonotic members of this genus are known to circulate in other mammals, such as pangolins [36,48,49,50,51]. Although direct zoonotic transmission of HPIVs to humans is rare, wild and domestic animals, including rodents, primates, and sometimes domestic dogs, may serve as secondary hosts or reservoirs for related viral strains [36,48,49,50,51]. The genetic diversity within respiroviruses indicates that cross-species transmission events, while uncommon, could potentially arise in contexts involving close human–animal interactions.

RETRACTED

Morbilliviruses, including MV, CDV, and Cetacean morbillivirus (CeMV), exhibit a complex relationship with their hosts. MV is an exclusively human pathogen, closely related to the now-eradicated rinderpest virus (RPV), which was a significant pathogen in cattle [85]. It is widely believed that measles emerged from a cross-species transmission event from cattle to humans, although the exact direction of this spillover has not been definitively established [86]. The timeline for when measles became endemic in human populations remains uncertain, but if MV originated from cattle, its emergence would be constrained by the divergence between MV and RPV. Molecular clock studies estimate this divergence occurred as early as the late 9th century [87,88]. CDV affects a wide range of terrestrial carnivores, including domestic dogs (*Canis lupus familiaris*), lions (*Panthera leo*), ferrets (*Mustela putorius furo*), and various wild carnivores [52]. CeMV primarily infects marine mammals, such as dolphins (*Delphinidae*) and whales (*Balaenopteridae*), causing significant outbreaks, with potential spillover risks to humans involved in marine mammal rehabilitation or handling activities [53].

### 3.2. Ecological Changes and Anthropogenic Factors

Although the risk of spillover from wildlife to humans has been linked to ecological changes and anthropogenic factors, the underlying mechanisms remain unclear [89]. The integrity of natural habitats plays a crucial role in maintaining the balance between wildlife populations and zoonotic disease dynamics. However, human-driven habitat alterations, particularly deforestation, agricultural expansion, and urbanization, have significantly disrupted this balance [2,90]. These changes displace wildlife, forcing them into closer proximity with human populations and domesticated animals, thus creating new opportunities for viral spillover [91]. For example, NiV virus outbreaks in Southeast Asia have been linked to habitat changes that drove fruit bats to forage in cultivated areas near pig farms, enhancing transmission pathways to humans [92]. In 2011, an outbreak of NiV was reported in northern Bangladesh, resulting in 15 deaths [93]. Subsequent research indicated that the primary mode of NiV transmission in Bangladesh is the consumption of infected raw date palm fruits [94]. These findings suggest that potential future outbreaks of NiV may be associated with habitat changes that prompt fruit bats to forage in agricultural areas, thereby increasing potential transmission pathways to humans [92]. Habitat fragmentation reduces biodiversity, which can exacerbate disease emergence risks. High biodiversity typically provides a “dilution effect”, interrupting pathogen transmission [95]. As ecosystems degrade, the remaining species—often adaptable to human environments—become more concentrated, increasing pathogen transmission likelihood [95]. This is evident in Australia, where land-use changes have heightened contact between flying foxes and human communities, leading to recurrent Hendra virus spillovers [96]. Additionally, intensive livestock farming near wildlife habitats could contribute to the emergence and spread of zoonotic paramyxoviruses [97]. High-density livestock operations create ideal conditions for cross-species transmission, exemplified by the Nipah virus outbreak in Malaysia in 1998, where bats transmitted the virus to pigs, subsequently infecting humans [98].

RETRACTED

The global wildlife trade also poses a considerable risk, facilitating the movement of potentially infected animals across borders. Live animal markets, where diverse species are housed in close quarters, have been linked to several zoonotic disease outbreaks [99]. The trafficking of bats and other *paramyxovirus* reservoirs increases the likelihood of spillover events into new species, including humans [99]. Rapid urbanization and increasing human mobility further expand the geographical reach of zoonotic paramyxoviruses [100]. Urban sprawl encroaches on natural habitats, enhancing human–wildlife interactions, while global travel allows pathogens to spread rapidly across continents [100]. Given the complex interplay of zoonotic, ecological, environmental, and anthropogenic factors, the implementation of a “One Health” approach is critical. This integrative strategy recognizes that human health is closely linked to the health of animals and ecosystems, and thus, interdisciplinary collaboration is essential to address the root causes of zoonotic disease emergence. By fostering collaboration across public health, veterinary science, environmental conservation, and agricultural sectors, the One Health approach aims to improve disease surveillance, enhance early detection of spillover events, and implement preventive measures that reduce habitat destruction and manage wildlife interactions [101,102]. For instance, recent studies have highlighted that integrated health strategies involving wildlife conservation and land-use planning can reduce the risk of zoonotic disease outbreaks, thus supporting both human and environmental health [102]. Understanding the interplay of ecological, environmental, and anthropogenic factors is vital for predicting and mitigating zoonotic risks [103] (Figure 2). Addressing these interconnected issues—by reducing habitat destruction, improving wildlife monitoring, and regulating wildlife trade—is essential to prevent future outbreaks and safeguard both human and animal health [103].

RETRACTED

## 4. Transmission Mechanisms and Pathogenesis

### 4.1. Molecular Mechanisms of Cross-Species Transmission

The mechanisms by which zoonotic paramyxoviruses overcome cross-species barriers and establish infections in new hosts remain a critical area of investigation [20,23]. Cross-species transmission is facilitated by a combination of molecular adaptations in the virus and ecological conditions that increase contact between different host species. At the molecular level, a primary factor in host-switching is the interaction between viral RBPs and host cell receptors [104]. The viral receptor specificity guides not only its ability to infect a new species but also the tissue tropism within the host, which can influence disease severity and transmission potential [39,105]. Among zoonotic paramyxoviruses, RBPs share common structural features with six-bladed β-propeller domains [104]. Viruses with HN proteins bind to sialic acid residues on host cells, such as respiroviruses [106]. In contrast, those with H or G proteins attach to host surface proteins such as henipaviruses, pararubulaviruses, and morbilliviruses [107,108,109,110]. However, little is known about how often and in what circumstances viral adaptation may occur within the host [111].

Henipaviruses exploit highly conserved ephrin receptors for cell entry, increasing the likelihood of cross-species spillover. NiV and HeV utilize ephrin-B2 (EFNB2) to facilitate a wide range of host infections, such as bats, pigs, horses, dogs, and humans. Additionally, these can use ephrin-B3 (EFNB3) as an alternative receptor [107,112,113]. EFNB2 is expressed in neurons, endothelial cells, and smooth muscle within arterial vessels, which correlates with the tissue tropism and pathological features of NiV and HeV infections in humans. EFNB3, primarily expressed in the central nervous system (CNS), shows both distinct and overlapping expression with EFNB2, enabling NiV and HeV to infect the CNS and cause severe encephalitis [39,114]. Given the significant conservation of ephrin receptors, emerging henipa-like viruses that utilize these receptors are likely to require minimal adaptation to enter and infect human hosts.

For viral entry, morbilliviruses utilize two key receptors, (i) the signaling lymphocytic activation molecule (SLAMF1/CD150) and (ii) the nectin-4 antigen, for entry into immune and polarized epithelial cells, respectively [110,115,116]. SLAMF1 shows a significant degree of variation in amino acid sequences across species, while nectin-4 remains relatively conserved. These species-specific differences in SLAMF1 have driven the evolution of morbillivirus RBPs, leading to reduced efficiency in recognizing SLAMF1 from hosts other than their natural reservoirs [109]. As infection of immune cells in the upper respiratory tract is crucial for initiating productive infections, the limited ability to bind “foreign” SLAMF1 is thought to restrict cross-species transmission of morbilliviruses [110,117]. After extensive SLAMF1-dependent replication in lymphoid tissues, the virus then utilizes nectin-4 for exit, infecting lung epithelial cells from the basolateral side, facilitating viral shedding into the airways [116]. Despite its high conservation, nectin-4 alone is not considered a significant factor in driving morbillivirus spillover. An exception to the typical species restriction of morbilliviruses is the CDV, which exhibits an unusually broad host range, infecting a wide variety of carnivores and even some non-carnivorous species [109,118]. CDV has also spilled over into non-human primates, leading to outbreaks of lethal disease [119]. Notably, only a few mutations in the RBP of CDV are sufficient to enhance the recognition of human SLAMF1 [120,121,122]. Given CDV’s ability to adapt to human SLAMF1, there is concern that unvaccinated humans could potentially serve as hosts for this virus [109]. Vaccination against the MV is recognized to confer cross-protective immunity against various other morbilliviruses [123]. Consequently, sustaining measles vaccination initiatives within the population, even after the eradication of MV, could be highly valuable in preventing potential zoonotic morbillivirus outbreaks [109]. Metagenomic studies have identified morbillivirus RNA in bats, *Myotis bat morbillivirus* (MBaMV), which was detected in a *Myotis riparius* bat, and PBZ-1381, found in a *Phyllostomus hastatus* bat [66,124]. Employing a reverse genetics approach, Ikegame and colleagues [125] have demonstrated that MBaMV preferentially uses Myotis SLAMF1 and possesses relatively poor usage of human SLAMF1. Structural analysis of MBaMV’s RBP showed that is likely incapable of forming two of the three critical salt bridges that facilitate interaction between the MV RBP and SLAMF1 in human species [126,127]. In contrast, PBZ-1381 appears to be more compatible with human SLAMF1, as a single-point mutation could restore the missing salt bridge [126,127]. These findings imply that, like the canine distemper virus (CDV), PBZ-1381 may require only a few mutations to adapt to and utilize human SLAMF1 [66,124].

RETRACTED

Pararubulaviruses, even if they are phylogenetically related to sialic acid-dependent orthorubulaviruses, exhibit notable differences in their RBP sequences. Specifically, pararubulaviruses lack the conserved sialidase hexapeptide motif ’NRKSCS’, which is characteristic of paramyxoviruses that utilize sialic acid for cell entry [128,129]. Molecular studies have confirmed that several pararubulaviruses, including MenV and Sosuga virus SosV, do not depend on sialic acid for host cell entry [128,129,130]. Among the pararubulaviruses identified to date, only the receptor-binding protein of Achimota virus 2 (AchiV-2) retains all seven conserved residues typically associated with the sialic acid active site; however, none of the known species possess the complete sialidase hexapeptide motif [131]. This strongly suggests that pararubulaviruses utilize protein-based receptors. These receptors are likely highly conserved across mammalian species, as pararubulaviruses have been found to naturally infect bats, pigs, and humans without requiring specific adaptations in their RBPs. Experimental infections in pigs (MenV), bats (SosV), and small mammals such as guinea pigs and ferrets (AchiV-1 and AchiV-2) have demonstrated that viral replication primarily occurs in the small intestines and secondary lymphoid organs [108,132,133]. Since tissue tropism across species is maintained, the receptor is probably conserved within this genus. Therefore, to understand the zoonotic potential of emerging pararubulaviruses, the identification of host receptors is pivotal.

The primary receptors for respiroviruses are sialic acid-containing glycoconjugates, which are abundantly present on the surface of host epithelial cells, particularly in the respiratory tract [134]. The HPIVs, key members of this genus, bind to these sialic acid residues via their hemagglutinin-neuraminidase (HN) glycoprotein [134]. This dual-function protein facilitates viral attachment to the host cell by recognizing and binding to sialic acids, and it also cleaves these residues during viral release to prevent self-aggregation [134].

### 4.2. Viral Replication and Immune Evasion

After viral attachment, the F glycoprotein triggers the fusion of the viral and host cell membranes, enabling the viral RNP to enter the cytoplasm [135]. The RNP serves as the template for the viral RNA polymerase complex comprising the P and L proteins. This complex initially functions in transcription, synthesizing viral messenger RNA (mRNA) from the RNP template [135]. The polymerase complex switches roles during replication, synthesizing full-length complementary positive-sense RNA (+RNA), which is then replicated into new RNP complexes [135]. These (−RNPs) are ultimately packaged into progeny virions. Both transcription and replication occur in virus-induced inclusion bodies within the cytoplasm [136,137]. In the later stages of infection, the newly formed RNP complexes and other viral proteins are transported to specific areas of the plasma membrane, where they contribute to the assembly and budding of new viral particles [138].

RETRACTED

Beyond receptor compatibility, successful spillover requires that the virus be capable of efficiently replicating within the host’s cells [139]. After entry, the virus must navigate the cellular environment, co-opting host machinery for viral replication while avoiding detection and suppression by the innate and adaptive immune system [140,141]. While numerous zoonotic viruses are adept at exploring a wide variety of potential hosts, mere entry into a host cell does not guarantee effective replication and dissemination. Not all cells provide an environment conducive to viral replication; specific host factors can either facilitate or impede the viral life cycle. Once inside the host cell, intrinsic immunity and antiviral restriction factors can significantly impair viral replication and attenuate secondary transmission [20,142]. To evade these host-antiviral defenses, paramyxoviruses typically express, often species-specific, accessory proteins that antagonize host innate immune responses, facilitating immune evasion [28]. The P gene, via RNA editing or overlapping ORFs, produces several products, such as C, V, and W accessory proteins, that play a critical role in viral immune evasion. These proteins act as key antagonists of type I interferon (IFN-I) production and other antiviral responses of the innate immune system [26,27,28]. Interferons activate a variety of antiviral genes that inhibit viral replication and spread, making suppression of this response essential for successful infection. Additionally, some viruses, such as *Orthorubulavirus*, encode small hydrophobic (SH) proteins that inhibit NF-κB signaling, a key regulator of immune and inflammatory responses. This suppression of immune pathways enhances viral persistence within the host [26,27,28]. Henipaviruses, including Hendra and Nipah viruses, exhibit a high degree of immune evasion and efficient replication following host entry, contributing to the severe and often fatal outcomes associated with human infections [38]. In particular, the henipaviruses produced proteins particularly effective at antagonizing human toll-like receptor and interferon signaling pathways, contributing to their pathogenicity during spillover events [143,144]. For instance, NiV is unable to induce encephalitis in wild-type mice, but infection in IFNAR knockout mice leads to neurological disease, emphasizing the virus’s limited capacity to counteract the mouse immune system [145,146,147]. Cedar virus (CedV), which lacks V and W proteins, does not cause disease in small-animal models, further underscoring the role of these proteins in pathogenicity [148]. Its non-pathogenic nature is largely due to its failure to inhibit host antiviral defenses [148,149] and its inability to utilize ephrin B3 as an entry receptor [150,151]. However, the fusion capabilities of CedV glycoproteins have not yet been fully explored and may also play a role in its reduced pathogenicity [152]. Since sialic acid molecules are highly conserved across species, it would be expected that paramyxoviruses utilizing sialic acid as a receptor would have a higher propensity for cross-species transmission. However, there have been no significant outbreaks of sialic acid-dependent paramyxoviruses spilling over from animals to humans, indicating potential post-entry barriers in new hosts. For instance, while HPIV-3 and bovine parainfluenza virus 3 (BPIV-3) are both antigenically and genetically similar, BPIV-3 exhibits reduced replication in humans, whereas HPIV-3 can cause disease [153]. These observations highlight the importance of post-entry compatibility, particularly involving viral accessory proteins, for successful infection in new hosts [20].

RETRACTED

## 5. Epidemiological Risks and Public Health Impact

The global public health community is particularly concerned about the possibility of novel, highly transmissible *paramyxovirus* strains emerging with pandemic potential [1,2]. These viruses have shown a propensity for rapid adaptation and evolution in new hosts, and their high mutation rates increase the likelihood of producing more virulent or transmissible strains, similar to what has been observed with other RNA viruses like SARS-CoV-2 [57,73,74,75,76]. Historically, outbreaks of zoonotic paramyxoviruses have been localized but severe. For instance, the NiV outbreaks in Malaysia and Bangladesh in the late 1990s and early 2000s were associated with widespread respiratory disease and encephalitis, with limited human-to-human transmission [154]. However, there is growing concern that with increased global travel and urbanization, future paramyxovirus outbreaks may not remain confined geographically. If a highly transmissible strain were to emerge, particularly one capable of sustained human-to-human transmission, the global consequences could be catastrophic [103]. The public health implications of a pandemic caused by a novel paramyxovirus would be profound, particularly given the limited treatment options available [155]. There are no licensed vaccines for human NiV infection or many other paramyxoviruses, and antiviral therapies remain largely experimental [155,156]. Moreover, the respiratory and neurological symptoms associated with these infections could overwhelm healthcare systems, especially in resource-limited regions [34]. The potential for such viruses to cause widespread social and economic disruption on a global scale underscores the need for urgent investment in preparedness measures, including enhanced surveillance, development of vaccines, and global collaboration to identify and mitigate emerging zoonotic threats. The increasing frequency of zoonotic spillovers, coupled with environmental and societal changes, raises the alarming prospect of a future pandemic. Proactive measures are essential to avert the emergence of new, highly transmissible paramyxovirus strains that could pose a dire threat to global public health.

RETRACTED

## 6. Prevention and Surveillance Strategies

Emerging zoonotic paramyxoviruses pose a significant public health risk due to their ability to jump between species and cause severe outbreaks in humans and animals. Preventive measures and robust surveillance systems are critical in mitigating the impact of these viruses. This section outlines key strategies for preventing zoonotic transmission and improving surveillance to detect and respond to potential outbreaks. The increasing overlap between human activities and wildlife habitats has facilitated the emergence of zoonotic pathogens, including paramyxoviruses [23]. Therefore, enhanced surveillance at the wildlife–human interface is essential for early detection and prevention of viral spillovers [157]. Bats, in particular, serve as natural reservoirs for many paramyxoviruses, including henipaviruses and pararubulaviruses [158]. Establishing long-term monitoring programs to track changes in bat populations, their migration patterns, and rates of viral shedding is crucial. These efforts should be focused on high-risk areas where human and livestock interactions with bats are common, particularly in regions undergoing deforestation, urbanization, or agricultural expansion. Routine collection and genetic sequencing of viral samples from bats and other potential hosts, such as pigs and horses, can provide valuable insights into viral evolution and the likelihood of spillover events. The use of advanced genomic tools can aid in identifying novel paramyxoviruses and tracking mutations that may enhance their zoonotic potential [159]. In order to maximize the effectiveness of these surveillance efforts, it is vital to adopt a One Health approach. This approach integrates veterinary, environmental, and human health sectors, promoting collaboration among field ecologists, veterinarians, epidemiologists, and public health officials [102]. Such a collaborative framework facilitates data sharing and allows for more comprehensive risk assessments, thereby strengthening the overall capacity to mitigate the emergence of zoonotic paramyxoviruses.

RETRACTED

Strengthening diagnostic capacities is essential for controlling zoonotic outbreaks caused by paramyxoviruses, particularly in low-resource settings where these viruses are likely to emerge and where diagnostic capacities are often inadequate. Investing in rapid diagnostic tools, such as point-of-care PCR tests and antigen detection kits, is crucial for early detection in both humans and animals. These tools must be easy to deploy in the field, especially in regions with limited access to centralized laboratories. Establishing regional diagnostic networks can improve sample sharing and capacity-building efforts, while also prioritizing the training of local healthcare professionals and veterinarians in sample collection, viral detection, and reporting procedures. Given the broad host range of many paramyxoviruses, developing cross-reactive assays that can detect multiple species of the virus, including novel variants, would significantly enhance surveillance capabilities [160]. These tests should also be designed to differentiate between closely related viruses such as Hendra and Nipah.

Proactive vaccination and antiviral strategies are crucial for preventing the spread of zoonotic paramyxoviruses, particularly in high-risk human and animal populations. Vaccinating livestock and companion animals that may act as intermediate hosts for paramyxoviruses is an effective preventive measure; for example, vaccination campaigns against Hendra virus in horses have proven successful in Australia, reducing the transmission risk to humans [161]. Similar strategies should be considered for other species at risk of paramyxoviruses infection. While there are currently no vaccines for most zoonotic paramyxoviruses, research and development in this area are essential, with a focus on henipaviruses, particularly Nipah virus, due to its high mortality rate. Research into broad-spectrum vaccines that could protect against multiple paramyxoviruses could also provide a long-term solution. Additionally, the development of antiviral therapies targeting key stages of the paramyxoviruses’ replication cycle could offer therapeutic options during outbreaks. Host-directed therapies that modulate immune responses may be promising, especially in mitigating the severe immune-mediated damage seen in diseases like Nipah virus.

RETRACTED

## 7. Conclusions

In conclusion, zoonotic paramyxoviruses, particularly those within the Henipavirus and Pararubulavirus genera, pose an increasing global public health threat due to their ability to cross species barriers and, in some cases, cause severe disease in both human and animal populations. This review has underscored the critical role played by bat species as key reservoirs for these viruses, with henipaviruses like Hendra and Nipah demonstrating the devastating consequences of zoonotic transmission, marked by high mortality rates and significant socioeconomic impacts. In contrast, pararubulaviruses, while generally associated with milder or asymptomatic infections in humans, still have the potential to cause disease and warrant closer surveillance. The molecular mechanisms that allow these viruses to jump between species—such as viral replication strategies, host receptor adaptations, and immune evasion tactics—remain a focal point of research. Understanding these mechanisms is crucial for identifying the factors that drive interspecies transmission, especially in the context of increasingly disrupted ecosystems and wildlife–human interfaces. Ecological factors, including habitat loss, urbanization, and shifts in bat population dynamics, are playing a major role in increasing the frequency of human–wildlife interactions, which in turn raises the likelihood of viral spillover events. In addressing the public health impact of emerging paramyxoviruses, this review emphasizes the urgent need for enhanced and coordinated surveillance systems that can detect zoonotic pathogens early, particularly in regions where human–wildlife contact is high. Strengthening diagnostic capacities, especially in low-resource settings where outbreaks are more likely to occur, is another crucial element in improving global preparedness. Furthermore, proactive vaccination strategies for both animals and humans, along with the development of targeted antiviral therapies, are necessary to prevent and control future outbreaks. By highlighting recent advancements and identifying key knowledge gaps, this review serves as a call to action for further research aimed at deepening our understanding of zoonotic paramyxoviruses. Equally important is the need for robust public health policies that can support early detection, containment, and prevention efforts. As human populations continue to encroach on wildlife habitats, the potential for zoonotic spillovers will likely increase, making it imperative to prioritize the development of effective interventions that can safeguard both human and animal health.

RETRACTED

## Figures and Tables

**Figure 1:** Primary evolutionary theories involved in the generation of new emerging zoonotic paramyxoviruses with epidemic potential.

**Figure 2:** The ecological, environmental, and anthropogenic factors for predicting and mitigating zoonotic risks.

**Table 1:** Zoonotic paramyxoviruses, their hosts, geographical distribution, mortality rate, evolution rate, and epidemic potential risk.

Subfamily	Genus	Species	Primary Host	Spillover Hosts	Distribution	Mortality Rate	Evolution Rate	Epidemic Potential	Refs.
*Orthoparamyxovirinae*	*Henipavirus*	Nipah virus (NiV)	*Pteropus* fruit bats	Pigs, humans	South and Southeast Asia	40–75%	High	Moderate to high (human-to-human transmission)	[7,8,9]
		Hendra virus (HeV)	*Pteropus* fruit bats	Horses, humans	Australia	57% in humans, 80% in horses	High	Low to moderate (localized outbreaks)	[7,8,9]
		Langya virus (LayV)	Shrews	Humans	China	No deaths reported	Moderate	Low to moderate (few cases)	[10,11,19]
	*Respirovirus*	Human parainfluenza virus (HPIV 1-4)	Humans, zoonotic potential unclear	None	Global	Low mortality, mild in most cases	Low	Low (seasonal epidemics)	[36,48,49,50,51]
	*Morbillivirus*	Measles virus (MV)	Humans (potential zoonotic origin)	None	Endemic globally, vaccine-preventable	<1% (with care)	Low, established human pathogen	Low (controlled with vaccination)	[41,42,47]
		Canine distemper virus (CDV)	Domestic and wild canines	Humans (?)	Global in animal hosts	High in animals, rare in humans	Moderate	Low (rare zoonotic spillover)	[52,53]
		Cetacean morbillivirus (CeMV)	Cetaceans	Unknown (potential zoonosis)	Global in cetacean populations	Unknown in humans	Moderate	Low (potential zoonotic risk)	[53]
*Rubulavirinae*	*Pararubulavirus*	Menangle virus (MenV)	Fruit bats	Pigs, humans	Australia	Unknown in humans	Moderate	Low (rare zoonotic spillover)	[32,32]
		Sosuga virus (SOSV)	*Rousettus aegyptiacus* bats	Humans	Central and East Africa	Moderate illness, severity unknown	Moderate	Low (sporadic cases)	[14,33]
*Avulavirinae*	*Orthoavulavirus*	Newcastle disease virus (NDV)	Wild birds, poultry	Humans	Global in birds, poultry exposure	Low, mild, self-limiting infections in humans	Moderate	Low (rare zoonotic cases)	[30]
